# Nutritional status, antioxidant activity and total phenolic content of different fruits and vegetables’ peels

**DOI:** 10.1371/journal.pone.0265566

**Published:** 2022-05-12

**Authors:** Yumna Sadef, Tayyaba Javed, Rimsha Javed, Adeel Mahmood, Mona S. Alwahibi, Mohamed S. Elshikh, Mohamed Ragab AbdelGawwa, Jawaher Haji Alhaji, Rabab Ahmed Rasheed

**Affiliations:** 1 College of Earth and Environmental Sciences, University of the Punjab, Lahore, Pakistan; 2 Department of Environmental Sciences, GC Women University Sialkot, Sialkot, Pakistan; 3 Department of Botany and Microbiology, College of Science, King Saud University, Riyadh, Saudi Arabia; 4 Genetics & Bioengineering, Faculty of Engineering and Natural Sciences, International University of Sarajevo, Sarajevo, Bosnia and Herzegovina; 5 Department of Health Sciences, College of Applied Studies and Community Service, King Saud University, KSA, Riyadh, Saudi Arabia; 6 Histology & Cell Biology Department, Faculty of Medicine, King Salman International University, South Sinai, Egypt; Ghazi University, PAKISTAN

## Abstract

The present study assessed nutritional status, antioxidant activity, and total phenolic content in fruits, i.e., mango (*Mangifera indica*), apple (*Malus domestica*), and vegetable, i.e., bottle gourd (*Lagenaria siceraria*), and ridge gourd (*Luffa acutangula*) peels. The antioxidant activity and total phenolic content (TPC) were evaluated by using methanol extracts along with 2, 2-diphenyl-1-picrylhydrazyl (DPPH), Folin–Ciocalteu (FC) assay, respectively having Butylated hydroxytoluene (BHT) and Gallic acid (GA) as standard. The TPC and antioxidant activity in the peels ranged from 20 mg GAE/g to 525 mg GAE/g and 15.02% to 75.95%, respectively, which revealed that investigated fruit and vegetable peels are rich source of phytochemical constituents. Bottle gourd peels exhibited the highest value of DPPH compared to the rest of the peels included in the study. Likewise, mango peels had the highest TPC as compared to the rest of the fruit peels. This research showed that the utilization of agricultural wastes should be promoted at commercial level to achieve the nutritional benefit at zero cost and minimize the generation of biological waste.

## Introduction

High-valued commercial crops such as fruits and vegetables are a vital subsector within agriculture. The development of fruits initiates from ovaries-specific tissues of the flower, or some additional tissues [1]. The presence of certain bioactive compounds containing nutritive and non-nutritive property such as, electrolytes, minerals, vitamins, fat, carbohydrates, dietary fiber, proteins, energy, and polyphenols like phenolics, and flavonoids are enriched in fruits and vegetables [2–4]. Many of these multifunctional compounds are reported to have strong correlation with decreased morbidity and mortality in humans from many devastating infectious and chronic illnesses [5]. Polyphenols are essential in the daily diet of human. Subsequently, they inhibit oxidative damage to cells triggered by reactive oxygen species (ROS), causing severe health issues such as atherosclerosis, rapid aging, and cancer. Antioxidants activity of polyphenols present in fruit peels could treat serious diseases [6, 7]. Phenolic compounds and pigments are the primary groups of compounds that contribute to the antioxidant activity of vegetables, fruits, cereals, and other plant-based materials.

Kalpna and Mital [8] reported that polyphenols are natural antioxidants that act as scavengers and inhibitors of free radicals responsible for oxidative damages to both the fruits and vegetables (their primary purpose) and human body (via intake of fruit and vegetables). The plant defense mechanism is stimulated due to antioxidant expression of polyphenols [9–11]. Presence of other essential compounds such as calcium and certain beneficial nutrients like vitamins in fruit and vegetables has further been suggested to prevent osteoporosis in adults to stimulate better health and strong bones [12]. Therefore, availability of phytochemicals in the human diet is a potential contributor towards substantial health, ultimately preventing from various diseases [13]. Southon et al. [14] reported that fruits are more enriched with nutrients than vegetables. The World Health Organization (WHO) board on nutrition, diet and inhibition of chronic diseases suggested daily intake of fruits and vegetables should not be less than 400 grams for healthy life [15].

Pakistan has significant production of fruits and vegetables; however, a large portion of the fruits and vegetables is dumped as waste [16]. *Malus domestica* commonly known as apple, member of the Rosaceae family, is widely consumed by human. It is beneficial to human health due to the presence of numerous biologically active compounds like monosaccharides, minerals, dietary fiber, and phenolic contents. These compounds play a crucial role in antioxidant functioning and are present in significant concentrations in apple peels as compared to flesh [17, 18]. Therefore, apple peel is rich source of nutrition for human diet as it provides resistance to various diseases [19]. Mango (*Mangifera indica)*, belonging to the flowering plant family Anacardiaceae and *Mangifera* genus, is among the world’s highly attractive and well-consumed tropical fruits [20]. It is rich in fiber, vitamins A, B, C, protein, energy, minerals, carbohydrates, proteins, fats, and phenolic compounds. These compounds provide strong scavenging ability, promote immune modulation, anti-lipid peroxidation, cardiotonic improvement, reduce hypotensivity, improve wound healing, counter-degenerative and anti-diabetic activities all of which are crucial benchmarks for better growth and development of the human body [21].

Agrawal et al. [22] demonstrated that Cucurbitaceous family usually called cucurbits contains various vegetable gourds, i.e., *Lagenaria siceraria* (Molina) Standley. The plants in this family are of medium size, including 118 genera and 825 species, all of which are widespread in the hot climatic regions of the world. These species are among the earliest cultivated plants used for medicinal and nutritional purposes. Bottle gourd (*Lagenaria siceraria*) is one of the most commendable vegetables because of high vitamin B content, fair vitamin C and phenolic content, and choline. It is considered an imperative source of beta-carotene, ascorbic acid, vitamin B complex, carbohydrates, pectin and dietary soluble fibers, minerals, amino acids, and other vitamins. It also contains phenolic acids, phenolic acid glycosides, terpenoids, flavonoids, and other vital oils [23]. *Luffa acutangula* is known as ridge gourd, has great importance for its ethnomedicinal properties and widely used in most of the Asian countries. Like apple and mango peels, bottle and ridge gourd peels are also highly nutritious and contain many beneficial bioactive compounds.

Baiano et al. [24] revealed that only households produce about 42% of the fruit/vegetable waste, another 38% is produced in the food processing industry, while the remaining 20% is produced in other parts of the food chain. Food waste generated from both households and food processing industries comprises of 50% of fresh fruit and vegetable peels, which are destroyed mechanically. These waste peels contain a high amount of phenolic content, proteins, lipids, fiber, carbohydrates, and energy that are responsible for their antioxidant activity and high nutritional value. Due to the presence of a variety of bioactive constituents, especially phenolic content, medicinal use and biological activities, fruit and vegetable peels are of great scientific interest and potential food.

The substitution of synthetic food antioxidants by natural ones has emerging trend in research on fruit and vegetables nutrition. Therefore, studies have been focused on plant-derived natural antioxidants in the recent decades [25]. The present study was aimed at determining the nutritional composition, total phenolic content, and antioxidant potential of fruits (apple and mango), and vegetables (bottle and ridge gourd) peels.

## Materials and methods

### Selection and collection of material

Apple, mango, bottle gourd and ridge gourd samples were collected from the local market of Lahore, province of Punjab, Pakistan (31.5204° N, 74.3587° E. Samples were sealed in polyethen bags, transported to the laboratory, and stored at 4°C until analysis. Random sampling technique was employed for sample collection.

### Preparation of peels powder

All samples were washed with deionized water to remove visible dirt. Samples were weighed and peeled using scraper. About 200 g of each fruit and vegetable peels were obtained from 1 kg of each sample. Peels were subsequently dried in a conventional hot air-drying oven at 50–70°C for 24–36 hours. After drying peels were homogenously mixed to a fine powder by mortar and pestle, stored in airtight jars and preserved at 4°C until use for solvent extraction.

### Nutritional analysis

The 5 g sample was dried at 105°C to a constant weight for determining the moisture content. of The ash, proteins, lipids, and crude fibers were analyzed according to AOAC methods [26], while carbohydrate content was determined by subtracting the percentages of moisture, ash, crude lipids, crude proteins, and crude fibers from 100 as described by Aina et al. [27].


Carbohydrate(%)=100–(%moisture+%protein+%ash+%lipids%+%crudefiber) (1)

Gross energy content was calculated by using the following formula, as described by Mukhtar et al. [18].


Energy(kcal/100g)=(%protein×4)+(%carbohydrate×4)+(%fat×9) (2)

### Preparation of peel extracts

The fruits and vegetables’ peels were prepared by following the method of Vasco et al. [28]. A total 2 g of each fruit and vegetable peel was extracted with 20 ml of 80% methanol, and 80 ml distilled water. The mixture was centrifuged at 3000 rpm for 10 min and the resulting supernatant was collected for further analyses.

### Qualitative analysis of antioxidant activity by DPPH assay

The qualitative antioxidant activity was assayed using 1, 1–diphyenyl, 2-picrylhdrazyl (DPPH) as described by Nithya et al. [29]. A total 50 μl of test sample was placed in a micro-Petri dish along with 100 μl of 0.1% methanol and DPPH. The mixture was incubated for 30 minutes in dark. After incubation, the test sample was evaluated visually for color transformation from purple to yellow or pale pink. By reacting with antioxidant, the stable free purple-colored 1, 1-diphenyl 2- picrylhydrazyl radical was reduced to yellow colored 2, 2-diphenyl-1-picrylhydrazyl.

### Quantitative analysis of antioxidant activity using DPPH assay

The antioxidant activity in terms of percent inhibition for peel extracts was determined using DPPH stable free radical assay easy. The 100 μl of the test sample was initially mixed with 2.7 ml of 0.1% methanol and then with 200 μl solution of 0.1% DPPH in methanol solution. Samples were then incubated for 30 minutes in the dark. Control samples containing the same amount of methanol and DPPH solution were also prepared. Subsequently, the absorption maxima of the solutions were measured using UV double beam spectra scan at 517 nm at 5-minute intervals. The percentage inhibition was then calculated using the following formula:

$$\%inhibition=\frac{Absorbance\;(control)–Absorbance\;(sample)}{Absorbance\;(control)}\times 100$$ (3)

The maximum antioxidant potential was found in bottle gourd and mango peels compared with the synthetic antioxidant butylated hydroxytoluene (BHT). The BHT is a chemical derivative of phenol (2, 6-di-tert-butyl-4—methylphenol) and acts as an antioxidant for the preservation of food as well as in pharmaceuticals, cosmetics, petroleum products.

### Determination of total phenolic content

Total phenolic content (TPC) was measured for the determination of antioxidant ability of fruit and vegetable peels by following the Folin-Ciocalteu (FC) method with slight modifications as described by Srinivas et al. [30]. Briefly, 0.5 ml of 10% Folin reagent was added to 0.1 ml of prepared extract. The mixture was then swirled and allowed to stand for about 6 minutes, followed by the addition of 1 ml of 7.5% Na_2_CO_3_ followed by thorough mixing. The resulting solutions could then stand for 2 hours at room temperature. After incubation, the absorbance was measured at 765 nm by using UV/Vis Shimadzu–Japan spectrophotometer. The calibration curve was obtained using gallic acid as standard with concentrations ranging from 100 to 1000 mg/ml. The results of TPC were expressed as gallic acid equivalent (GAE) per gram of dry sample concerning the gallic acid standard curve (R^2^ = 0.900). All samples were analyzed in triplicate and averaged.

### Statistical analysis

The descriptive statistics was determined using Statistica software. Correlations of the antioxidant activity and total phenolic content between fruits and vegetables extract samples were determined using Minitab version 17. One way ANOVA [31] and t-test was employed by Statistica software.

## Results and discussion

### Nutritional composition of fruit and vegetable peels

The nutritional composition of fruits and vegetables are presented in Table 1. The moisture content ranged from 8.81 ± 0.51% to 11.20 ± 0.31%. The highest moisture content was recorded for apple and ridge gourd peels (11–12%) and the lowest for in mango peels (8%). No significant differences were recorded among vegetables and fruits peels. The results obtained are comparable to earlier studies by Sogi et al. [32] and Leyva-Corral et al. [33]. Moisture content can be used as an index of the microbial stability and susceptibility to microbial contamination and degradation [34]. Apple and ridge gourd peels are highly susceptible to microbial degradation and require longer duration of time for drying.

**Table 1:** Nutritional composition (± standard deviation) of fruit and vegetable peels.

Sample	Moisture	Ash	Lipids	Fiber	Protein	Carbohydrates	Energy
	of total (%)	of dry matter (%)					kcal/100g
Mango	8.8 ± 0.51	3.5 ± 0.22	0.34 ± 0.05	4.5 ± 0.22	4.30 ± 0.05	78.5 ± 0.24	335 ± 1.2
Apple	11.9 ± 0.92	2.6 ± 0.52	0.18 ± 0.04	7.6 ± 0.06	1.24 ± 0.05	76.5 ± 1.4	313 + 6.0
Bottle gourd	9.9 ± 0.24	8.5 ± 0.27	0.15 ± 0.03	15.6 ± 0.20	12.2 ± 0.12	53.7 ± 0.85	264 ± 2.5
Ridge gourd	11.2 ± 0.31	7.3 ± 0.13	0.19 ± 0.02	17.6 ± 0.25	16.5 ± 0.18	47.3 ± 0.77	256 ± 2.1

Values are means ± standard deviations of three replicate measurements.

The ash content in fruit and vegetable peels ranged from 2.56 ± 0.52 to 8.52 ± 0.27% of dry matter. The lowest ash contents were noted in apple and mango peels and the highest in bottle and ridge gourd peels. Ash contents in the vegetables were significantly higher than fruits (p<0.050). The observed ash contents for the vegetable peels are significantly lower as compared to earlier reported studies, i.e., Saeed et al. [35]. While the percentage of mango and apple peels were 1.39 to 3.88% comparable to earlier observations by Ashoush and Gadallah [36] and Romelle et al. [37].

The lipid (fat) content ranged from 0.15 ± 0.025 to 0.34 ± 0.046% of dry matter. Bottle gourd peels had the lowest lipid content and mango peel had the highest lipid content. Aziz et al. [38] and Hung et al. [39] previously reported that lipid contents in apple and mango peels ranged from 0.1 to 0.32%. The lipid contents in vegetable peels recorded in our study were higher than reported those of Saeed et al. [35], who reported 0.18 ± 0.2% fat content in bitter gourd peels.

The crude fiber content and protein content ranged from 4.5 ± 0.22 to 17.6 ± 0.24% and 1.24 ± 0.045 to 16.52± 0.18% of dry matter, respectively. The vegetables had significantly higher contents of fiber (p = 0.050) and protein (p = 0.050) than fruits. The results indicated fruits and vegetables with higher protein content are more vulnerable to fungal degradation. Therefore, the overall results are consistent with those reported in Arumugam and Manikandan [40], who reported percentage of protein in mango as 4.27% which is lower compared to those observed by Saeed et al. [35], who reported 17.77 ± 1.8% fiber content and 20.37 ± 1.9% protein content in bitter gourd peels.

The carbohydrate content in the fruit and vegetable peels varied from 47.3± 0.76 to 78.5 ± 0.24% of dry matter. Fruit peels had significantly higher values of carbohydrate content as compared to vegetable peels (p = 0.050). This indicates that the fruit peels are potentially more useful for producing animal feed.

The energy contents ranged from 256 ± 2.08 to 335 ± 1.15 kcal/100g. The fruit peels had significantly higher values than vegetable peels (p = 0.050), possibly due to their different carbohydrate contents and minimum in ridge gourd peels. The results are slightly higher than Mukhtar et al. [18]. Energy content in apple fruits ranged from 37.6 to 73.28 kcal/100g.

### Inhibition (%)

Percentage inhibition of fruit and vegetable samples with BHT standard is shown in Fig 1. Results indicated that vegetables had greater scavenging potential than fruits.

**Fig 1:** Percent inhibition of different fruit and vegetable peels.

The percentage inhibition shown in fruits (apple and mango) was 67.27% and 73.16%, respectively, whereas for vegetables (bottle gourd and ridge gourd) it was 54.23% and 75.95%, respectively. The percentage inhibition in fruits and vegetables was compared with BHT, which was 77.12%. Comparison of percentage inhibition of fruits and vegetable peels with BHT indicated that minimum inhibition capacity was found in apple 29.11%, mango 34.28%, bottle gourd 34.12%, and ridge gourd 15.02%.

### Phenolic content

Phenolic contents have gained considerable interest because of their potential beneficial effects on human health. Phenolic contents have been reported to show antiviral, anti-allergic, antiplatelet, anti-inflammatory, anticancer, and antioxidant activities [41]. Quantification of total phenolic content in extracts of fruits and vegetables was carried out by using the Folin-Ciocalteau reagent. The TPC values were given in Fig 2.

**Fig 2:** Total phenolic content in fruit and vegetable peel extracts.

The total phenolic content ranged from 228 to 503 mg gallic acid equivalents (GAE)/g of fruit peel samples and 23 to 91 mg GAE/g of vegetable peel samples. On average, the two fruits had significantly higher phenolic content than vegetables (p = 0.05). This indicates that peels of the two fruits considered here may be used to produce natural antioxidant supplements in food and pharmaceutical industry.

## Conclusion

Food waste mostly fruits, and vegetable peel contains essential nutrients required for better human health. The present investigation showed that fruit peels are more nutritious for carbohydrates and contain significant amount of total phenolic content. This study focused on improving the extraction proficiency of polyphenols and antioxidants from fruits and development of strategies to utilize them in food and pharmaceutical manufacturing. This research showed that utilization of agricultural wastes such as fruit and vegetable peel waste should be promoted at commercial level. They are cost-efficient and organic-rich compounds having safe health benefits. Commercial preparations of natural fruits and vegetable peels to extract valuable bioactive components and to utilize them as a source of natural antioxidants support the basis of the present study as they are very high-value products, and their recovery can be economically attractive.
